# Analysis and Research on the Rehabilitation Effect of Physical Exercise on College Students' Mental Depression Based on Multidimensional Data Mining

**DOI:** 10.1155/2022/7656782

**Published:** 2022-07-13

**Authors:** Wen Zou

**Affiliations:** Chengdu Sports University, Chengdu, Sichuan 610041, China

## Abstract

In order to explore the physical exercise and psychological changes of college students, this study adopts the method of multidimensional data mining, taking 23,146 undergraduates from a university in Guangzhou, Guangdong Province, as the research object. On the basis of summarizing and analyzing the previous research literature, this study expounds the development background, current situation, and future challenges of multidimensional data mining technology. This paper introduces the methods and principles of sample selection and multidimensional assessment of the physical and mental depression of college students, analyzes the physical health status of college students, summarizes the psychological changes of college students before and after the intervention, and discusses the relationship between physical exercise and mental health of college students. In addition, this paper analyzes the influencing factors and psychological changes of college students' physical exercise and puts forward suggestions for improving the physical and mental health of college students. The results of this study show that with increasing age, college students have a lower risk of moderate anxiety and mild depression; girls are more prone to mild depression than boys; rural college students are more prone to mild, moderate anxiety; college students with nonmedical backgrounds were more likely to experience moderate anxiety than college students with medical backgrounds. During the intervention control period, continuous connection with others may encourage college students to actively use internal resources to actively cope with obstacles and setbacks, and as a protective factor, psychological resilience can appropriately weaken the association between risk factors in life and anxiety and relieve anxiety. The results of this study can provide a reference for further research on the physical exercise and psychological changes of college students.

## 1. Introduction

High infectivity and high risk are the main reasons for students to cause psychological problems such as fear, stress, and worry. Due to the concerns about their own health, coupled with the characteristics of today's media communication, spamming of information, especially the spread of rumors, has caused panic among college students and affected their psychological health [1]. The system data analysis module systematically processes and analyzes the results of the students' physical test data. After the query, it is displayed in a high-visibility form; the analyst can directly understand the students' specific physical health status based on the visual graphics, resulting in a sense of discomfort and threat. Due to the interaction and infection of emotions between individuals, the panic psychology and behavioral responses of some individuals often cause group panic [2]. On the other hand, it is difficult for the public to use the existing common sense and knowledge system to make rational judgments about the uncertain news of major public emergency events, which in turn leads to emotional instability and panic [3]. The intervention has hindered the opening of gymnasiums and other exercise venues, thereby limiting the conditions for college students to carry out physical exercise, and affecting the physical quality of college students to a certain extent [4].

Compared with traditional sampling and questionnaire surveys, data mining and algorithm analysis based on big data not only saves time, manpower, and material costs but also obtains a set of accurate and timely analysis and prediction results for each individual surveyed, achieving the maximization of personalization and pertinence of assessment [5]. Big data technology can realize data mining and algorithm analysis of college students' physical and psychological health. College administrators can grasp students' social status and learning status at any time, predict their psychological status, and pay close attention to high-risk students according to the results of algorithm analysis, and timely communicate with them [6]. Multidimensional data mining can analyze the number and time of college students entering and leaving the dormitory and the library according to the campus face recognition system. If the time to leave the dormitory is longer, the time spent in and out of the library is longer, and the time spent in the library is longer, it may indicate that students have less social interaction and study time [7]. Through this data model, information such as students' morning runs can be entered, and schools can observe students with weak physique in advance. Managers can obtain various data through more instruments and can process and analyze massive data in a timely manner, so as to more accurately grasp their own physical health and take effective improvement measures accordingly [8].

In order to explore the physical exercise and psychological changes of college students, this study adopts the method of multidimensional data mining and takes 23,146 undergraduate students from a university in Guangzhou, Guangdong Province, southern China, as research examples. On the basis of summarizing and analyzing previous research literatures, this study will expound the research status and significance of the impact on the physical and psychological health of college students, elaborate the development background, current status and future challenges of multidimensional data mining technology, introduce the methods and principles of sample selection and multidimensional assessment of college students' physical and mental depression, analyzed the physical health of college students before and after the intervention, summarize the psychological changes of college students before and after the intervention, discuss the relationship between physical exercise and psychological health of college students before and after the intervention, perform an analysis of the factors affecting the physical exercise and psychological changes of college students before and after the intervention, and finally propose the suggestions for improving college students' physical and psychological health under the intervention. The detailed chapter arrangement is as follows: Section 2 introduces research methods and data acquisition.  Section 3 is the results and its analyses.  Section 4 is the discussion.  Section 5 is the conclusion.

## 2. Research Methods and Data Acquisition

### 2.1. Sample Selection

This study adopts the method of multidimensional data mining and takes the undergraduate students of a university in Guangzhou, Guangdong Province, southern China, as an example to carry out the research on the physical exercise and psychological changes of college students before and after the intervention. This university has a total of 23,146 undergraduate students, including 13,915 males, 9,231 females, 5,984 freshmen, 5,823 sophomores, 5,691 juniors, and 5,648 seniors (Table 1). The spatiotemporal information knowledge map of college students' physical health psychological changes is to express the concepts, entities, attributes, events, etc. related to the intervention as triples, that is, subject, predicate, and object, using a resource description framework, and then establish each element, entity, the relationship between events, represented by a point-edge directed graph. The location attribute features change with time, and the event attribute changes with time; the spatiotemporal trajectory displays the trajectory path based on the map, and the time series events can be represented by the event axis view. The visualization of college students' physical health psychological changes adopts the node-edge method, through the switching and visual interaction of different spatial layouts such as force-guided layout, hierarchical layout, and ring layout, to discover the inheritance relationship and implicit laws between different college students' nodes.

School information management mainly includes a variety of management tools such as academic engineering system, educational affairs system, short message platform, and campus card system. These data can be collected together into a data center, and the problems existing in students can be summarized according to the corresponding data model, making the data self-practice to form expert models at all levels. If the time away from the dormitory is long, but the number of times in and out of the library is small and the stay time is short, it may indicate that the student has more time for social entertainment or class [9]. According to the analysis of the above situations, for students who are not active in social interaction and learning, managers can communicate with them in time. The prediction algorithm can not only analyze single data but also analyze multiple joint cross-data to obtain more accurate and detailed prediction results. It can not only analyze students' school information to achieve early warning but also try to analyze their smart phone search engine records, the usage of commonly used application software, social software chat records, and analysis of students' subconscious behavior and psychological state when playing games, etc. However, this data mining method needs to take into account the needs of application development and privacy security, so it can only be implemented under the protection standard and the establishment of relevant data security and privacy.

### 2.2. Multidimensional Assessment of College Students' Physical and Mental Depression Based on Multidimensional Data Mining

Multidimensional data mining can record students' personal information and physical and mental depression data such as body, psychology, vision, and physical examination results; multidimensional data mining can also combine third party physical and mental exercise auxiliary applications to monitor students' exercise in real time and use the multidimensional assessment method of physical and mental depression to evaluate students' physical and mental depression. The physical and mental depression exercise program can recommend different exercise programs for students and count the exercise and physical and mental depression of students in different student circles and conduct comparative analysis accordingly. Multidimensional data mining can support teachers to input personal and class information, check the physical and mental depression and changes of students in the class, and provide guidance and suggestions for students; it can also input personal and child information, check students' physical and mental depression and changes and add guidance suggestions [10]. The background system supports administrators to maintain user information, manage exercise programs, and comprehensively analyze the physical and mental depression of students; the data processing part can obtain real-time exercise data of students and conduct analysis and assessment, providing support for the data processing needs of different subsystems. Exercise plan refers to the designed exercise plan for body, mind, vision, and physical examination, and the administrator needs to set its attributes when adding exercise plan, such as category attribute and fitness attribute.  Figure 1 shows the multidimensional assessment model physical exercise and psychological changes of college students before and after the intervention.

College students' health data analysis and processing system based on big data can provide health management services for college students. The universities can understand students' physical health status through physical examination, build an interactively controllable basic service and medical ecological platform, and realize the interaction of key information between the system and the platform, so that colleges can provide students with efficient and personalized physical health services so as to promote the optimal management of students' self-health. Panic psychology is the main reason for irrational behavior, and the mechanism of forming panic psychology involves both individuals and information. On the one hand, the occurrence of major public crises often changes personal daily habits. Based on the age group interface, the analyst can also obtain the personnel data at each stage and the ratio of male to female students and use the method of inputting age to quickly find out the number and proportion of this age group. It contains multiple decision trees. The confusion matrix can be used to calculate the accuracy, specificity, and sensitivity of the model to evaluate the performance of the model. Big data analytics uses training data to build models that use relevant features and use fully trained models to make predictions on new data.

## 3. Results and Analysis

### 3.1. Psychological Changes of College Students before and after the Intervention

The study found that both male and female college students' health levels declined before and after the intervention, but the decline in male students was not as significant as the decline in female students. From the comparison of data under the influence of the intervention, the health level of male college students is higher than that of female college students. Female students' stress response is stronger than that of male students, and they account for a larger proportion. In addition, female students' anxiety level is generally higher than that of male students, and they will be the key population for psychological health in colleges in the future. In the face of this public health emergency, school management should take targeted intervention measures to reduce the group's overreaction to the intervention. In addition, the relevant education departments should also improve the physical exercise and psychological health education of students during the ongoing stage of the current intervention, especially giving more attention to the female group. As shown in Figure 2, college students who do not usually exercise after regular moderate-intensity physical exercise, the self-feeling of sleep has been greatly improved, and the percentage of the number of students who fall asleep for a long time has decreased significantly, indicating that had a long time to fall asleep after physical exercise have significantly shortened the time to fall asleep and become more likely to fall asleep. The general college students are changing to the direction of good sleep quality, and the sleep quality is changing to a better trend.

Classification models are based on known categories of data objects, while clustering is used to deal with unknown types of data objects. Clustering requires observational learning to divide the object set of physical health data into several similar object classes. Different clustering algorithms of college students' physical health big data also correspond to different standards such as division, level, density, grid, and model. These algorithms are suitable for understanding the impact of college students' study habits, living habits, and exercise habits on physical health. This kind of division is more scientific than the classification and observation based on traditional cognition, and it can also find the relationship between various data that could not be found in the past. Teachers personalize instruction for different groups. Such as students' courses, examinations, tests, learning, and assignments, the data types are diverse, including not only structured data such as study time and grades but also nonstructured data that are difficult to quantify such as learning assessment and teaching and social practice. The more the data is subdivided into each behavioral part, the more the characteristics of students' learning behaviors can be drawn, and the more objectively they can reflect the students' learning behaviors and then reflect the relationship between students' learning behaviors and physical health [11].

Due to students' isolation at home and receiving online physical education teaching, the teaching tasks and teaching objectives have undergone major changes, and the content of online physical education teaching has also been adjusted accordingly. Therefore, the content of online physical education should focus on life safety education, cognitive education on the connotation of sports principles, education on sports behavior norms, and education on physiological and psychological knowledge, so as to improve the quality of online physical education. At the same time, in the process of offline teaching, limited by the arrangement of class hours, the theoretical part of physical education teaching has a short teaching time and a long practical time. It is difficult to carry out a large number of practical teaching activities. Since it is difficult for online teachers to observe students' classroom performance, the focus of online teaching supervision in the classroom process determines the effect of physical education teaching [12]. At the same time, scientific and reasonable assessment and assessment can promote students' enthusiasm for learning and improve the quality of online physical education teaching. Students' satisfaction with online physical education courses is an important factor for students to actively build knowledge, and it is also one of the important indicators to test the teaching effect. Students recognize the online physical education course teaching, solve the difficulties in students' learning, and are inspired by it to acquire sports knowledge, so as to obtain higher satisfaction.

### 3.2. Physical Exercise of College Students before and after the Intervention

The severe situation has already had a certain degree of impact on the psychology of college students. The results show that the concentration, mood, temper, and mood of senior college students are more affected by the intervention, which is manifested in that college students' concentration in doing things decreases, their mood becomes unhappy, their mood becomes low, or they are easily excited. The reasons for the above changes may be that the off-campus internships, interschool exchanges, and other activities of senior college students have been seriously disrupted by the intervention, and the normal study plans of college students have been affected [13]. Parents who do not know much about the intervention are often prone to panic, and the psychological changes of parents will correspondingly affect the psychology of college students (Figure 3). The intervention will cause mental illness in college students to a large extent, and appropriate and effective psychological relief can relieve college students' psychological pressure and improve their bad psychological state. Physical exercise is a physical activity in which students choose suitable physical means to enhance their physical fitness and improve their spirits according to their own needs. Compared with before the outbreak, the proportion of girls with irregular work and rest is higher than that of male students. These changes may be more sensitive to male students than girls. In addition, there may be a lack of strict time control in schools in the home isolation area, and college students are prone to sleep problems.

Excessive media exposure may lead to a mix of too much correct and incorrect information, making it difficult for college students to find reliable sources of information and more at a loss, thus endangering their physical and psychological health. In addition, many college students express their negative emotions, such as fear, worry, tension, and anxiety, through social media, and these negative emotions are also spread through social networks [14]. Under the intervention, female students are more prone to mild depression than male students, and college students in rural and suburban areas are more prone to mild and severe anxiety and depression than urban college students. Based on different population characteristics and the responses of college students in emergencies found in this study, cross-institutional or community cooperation can be adopted to build different platforms to deal with information and adapt to different psychological adjustment needs. First of all, starting from media exposure, highly credible official information should be released in an efficient, fast, and transparent way to reduce unnecessary discussion and speculation among college students; secondly, school administrators are responsible for organizing online activities to enhance college students' sense of belonging and responsibility and social support, popularize psychological health knowledge, and carry out effective psychological monitoring of community college students.

The formation of public panic in major public emergencies comes from two aspects: individuals and information. In addition to the impact of external information on public psychology, the degree of attention and content of college students' attention to the event and the information processing and integration on this basis are the formation of psychology. In emergencies, crisis panic information will form emotional panic among college students in the process of network information dissemination. The intermingling of the thinking and opinions of the college students gradually forms an unorganized organizational force, and in these organizational forces, authoritative opinion expressers, and opinion leaders will be active. In the event of an outbreak, college students living off-campus experienced more mental stress than those who lived on campus, and their mental development was clearly visible: doubt, anxiety, safety, and regained confidence. Opinion leaders are active members of the group, with high influence, and often play a role in fueling or reversing the wind in the process of opinion dissemination and information transmission. The above studies all show that in major emergencies, college students tend to focus their attention on opinion leaders, and the degree of attention and core focus of college students on event-related information will affect their psychology and behavior.

## 4. Discussions

### 4.1. Relationship between Physical Exercise and Psychological Health of College Students before and after the Intervention

Modern psychological research shows that with the increase of exercise intensity, anxiety, tension, and depression and other adverse psychological states and emotions will gradually weaken with the consumption of physical functions and eventually reach a state of calm. During the quarantine period, compared with urban college students, rural college students have less corresponding learning equipment and immature network conditions at home. The daily routine, sleep, parent-child relationship, and going out of college students are all affected by the intervention. In the face of academic pressure, their concentration on work will also be reduced, and their mood will be relatively low. Epidemiological studies have shown that physical exercise can prevent or delay the onset of various mental disorders and has the effect of single or auxiliary treatment of college students' mental illness [15]. Physical exercise can improve the psychological health of college students by enhancing cognitive function; the cognitive-behavioral hypothesis also believes that physical exercise can induce positive thinking and emotion (Table 2). Exercise can positively affect the key areas of the brain and improve the mental and psychological conditions of exercisers. However, most of the current research results have explained and emphasized the exercise intensity, and moderate-intensity exercise suitable for exercisers is the premise of achieving good results. Therefore, college students should pay attention to the intensity and frequency of exercise when exercising, so as to avoid injury accidents caused by overdoing it.

College students feel more uncertain and uncontrollable when facing the intervention and some students may even have catastrophic thinking, exaggerating the consequences of the intervention, and then show varying degrees of psychological stress and even mental disorders. Some students will fall into fear, anxiety, anger and hostility, depression, sleep disorders, and physical discomfort, which makes it difficult to carry out treatment measures and has limited treatment effect [16]. The psychological emotions of college students during the intervention are complex and multilateral, and they are easily affected by the external environment. These may be the reasons for the anxiety and depression of college students living in rural areas. Sleep is closely related to the level of psychological health, and poor sleep quality is one of the factors that cause psychological problems. More than half of college students believe that they can avoid contracting the disease and the reason may be the formation of a fearless psychological defense mechanism in reverse. When all kinds of information about the spread of the intervention are overwhelming, students gradually realize that they have lost control of the intervention and use fear-relieving self-defense mechanisms. As each person's own health level is different, and the psychological processing mode of external emergencies is also different, the risk perception of crisis events will be different, resulting in different coping methods.

Physical ability refers to the ability of college students to unify their mind and body and coordinate and cooperate when they complete an activity. Compared with other abilities, it has certain particularity and is a combination of personality and physical and mental qualities composed of knowledge, technology, skills, and intelligence. Physical ability plays an important role in the cultivation of physical literacy. During the intervention, college students have strengthened their physical exercise by learning exercise knowledge, exercise methods, and exercise skills through the Internet. For the improvement of sports ability, most college students prefer onsite learning and onsite mutual exchanges, so that they can experience and learn sports skills and knowledge more intuitively. For physical education teachers, the teaching method of skills and knowledge is the teaching method adopted to reflect the performance of the body through the understanding of the students. Such offline guidance enables college students to learn with motivation and better mastery. During the intervention, many quarantined students are learning on line, during which, without the offline teaching guidance of teachers, it is inevitable that there will be discomfort during learning and it is necessary to systematically and gradually improve the Internet communication, as well as video production and communication skills. College students learn through the Internet, which is a new learning technology reform, which broadens the horizons of college students and enriches their cognition of physical skills mastery.

### 4.2. Analysis of Factors Affecting the Physical Exercise and Psychological Changes of College Students before and after the Intervention

The results of one-way analysis of variance showed that there was significant differences in the total score of psychological distress in the average monthly income of the family, and the more serious the psychological distress of college students from low-income families. As shown in Figure 4, the reason may be the uneven ratio of males and females in this study, and the fact that both rural and urban areas have strict control measures, screening standards, and isolation systems, which ensure the personal safety of the public and reduce the psychological burden of students. Although there is no difference in media exposure levels between the subjects in the severe areas and those in other areas, the risk of anxiety in the former is higher than that in the latter, indicating that college students in areas with severe situation face more severe psychological stress and more stress. Studies have shown that the higher the awareness of new coronary pneumonia, the lower the risk of mild anxiety among college students, the more comprehensive the understanding of new coronary pneumonia, the better the understanding of preventive measures, and the better their psychological state [17]. There are significant differences in the total score of psychological help in terms of age, gender, and average monthly income of the family. The possible reasons are that the psychological adjustment ability and troublesome problems of college students of different ages are different, and the needs of psychological help are also different. Female students are better at talking and are willing to seek social support, and psychological help-seeking attitude is more positive; compared with high-income families, low-income families have a more negative psychological help-seeking attitude due to objective factors such as economic conditions.

As shown in Table 3, with the increase of age, the risk of moderate anxiety and mild depression of college students is lower, which may be because the older the age, the more experience, the college students' social adaptability and psychological tolerance have improved. Therefore, colleges should pay attention to the psychological dynamics of young college students in a timely manner, maintain two-way communication through the Internet, and focus on providing crisis psychological support to junior college students. Female students are more prone to mild depression than male students, probably because female students are more emotional, relatively emotional, and easily infected by nervousness. Therefore, college psychological counseling centers should pay more attention to the psychological dynamics of female students and implement psychological intervention measures as soon as possible [18]. College students in rural and suburban areas are more prone to mild to moderate anxiety and mild to severe depression than urban college students. This may be due to the lack of basic medical resources in rural and suburban areas with the relatively weak public health prevention capabilities. College students with nonmedical background are more likely to have moderate anxiety than college students with medical background. College students with medical background have a complete biomedical knowledge reserve and have a more comprehensive understanding of COVID-19 related knowledge, while nonmedical background college students have relatively weak discrimination ability, it is easy for them to listen to rumors, and therefore, relevant departments should focus on health education for college students with non-medical backgrounds.

The findings of this study suggest that resilience plays an important mediating role between social support and college students' anxiety during COVID-19 control. Resilience has a positive effect on the generation and development of anxiety and leads to the relationship between social support and anxiety. During the intervention control period, continuous connection with others may encourage college students to actively use internal resources to actively cope with obstacles and setbacks, and as a protective factor, psychological resilience can appropriately weaken the association between risk factors in life and anxiety and relieve anxiety. Although the quarantine and prevention measures during the intervention control period have ensured the personal safety of returning college students, the consequent restrictions on freedom and delays in academic and research may lead to an increase in the risk of psychological distress. In this study, the psychological self-assessed health scores of college students before the outbreak and during the outbreak did not show significant differences. The possible reason is that the psychological assistance and health education of the society, colleges, and the support of family members played an important role. The second is that college students at home are worried that their psychological adverse reactions will bring bad consequences, so they show that they have a good psychological state, in order to be more easily accepted by teachers and classmates [19].

### 4.3. Suggestions for Improving the Physical and Psychological Health of College Students under the Intervention

According to the quality-stress theory of depression and the theory of bioecology, during the intervention, college students have different coping results due to their different perceptions of stressors and differences in quality, so the psychological quality of individuals is in the process of turning crisis into opportunity an important opportunity factor. The assessment of an individual's psychological quality is mainly carried out from three dimensions: cognition, personality, and adaptation. In terms of cognition, during the novel coronavirus pneumonia intervention, the psychological health status of medical college students was better than that of engineering and liberal arts college students, and their psychological health status was related to coping styles [20]. It can be seen that medical students have more protection knowledge due to their professional quality, and they have more reasonable cognition and response methods in the face of the intervention. During the prevention and control of new coronary pneumonia, the anxiety level of female college students is higher than that of male college students in five diagnostic indicators: anxiety, stress, sleep problems, cognitive problems, and depressive mood (Figure 5). In terms of personality trait differences, compared with other personality traits, individuals with neurotic personality are more likely to have negative emotions, and the personality toughness trait can alleviate the discomfort caused by life stress to the individual's body and mind.

College students of different grades have small differences in performance expectations and effort expectations, but subdividing the mean of each dimension, it can be found that the average performance expectations of college students in all grades are significantly lower than their average effort expectations. The mean value of college students' performance expectations gradually decreases. As far as grades are concerned, the mean value of effort expectations of college students in the third grade is significantly higher than the mean value of performance expectations of college students below the second grade, which indicates that college students with higher grades are more willing to make efforts to master systematic health knowledge [21]. As far as majors are concerned, there are significant differences in the effort expectations of different majors in the degree and method of teaching, but there is no significant difference in performance expectations. The scores of medical college students on performance expectations are significantly higher than those of nonmedical college students, indicating that medical college students believe that receiving systematic physical exercise is helpful for them to scientifically and effectively respond to public health crises. It also shows that medical college students are more willing to accept systematic physical exercise to deal with public health crises. There are no significant differences in performance expectations, effort expectations, and convenience conditions among college students of different gender stages, but only in social influence.

During the intervention, the psychological health level of college students living in rural areas was low, and they were prone to depression and anxiety. Because of the lack of basic medical resources and living materials in rural and suburban areas during the intervention, even some rural economies were affected. At the same time, the public health prevention awareness of most students in rural areas is weak, and there are many students who are disgusted and resist intervention prevention measures such as wearing masks due to the restrictions on folk customs. With the rapid spread of the intervention and the increase in online reports, college students gradually realized the seriousness of the virus, coupled with concerns about their own health, shortage of intervention prevention materials, and panic spread among students. Compared with the national norm, the sleep quality of college students is poor. The results of this study also pointed to the poor psychological health of students who fall asleep late and have short sleep duration [22]. The time to fall asleep and the duration of sleep are important factors that affect the level of psychological health. When the external environment is monotonous and constrained, college students are more likely to become dependent on mobile phones. The intervention involves a long period of home study, and students have a long time to control themselves; and there are few entertainment activities at home, and the use of mobile phones and computers is also longer than usual, and it is normal to fall asleep late. Therefore, the sleep and psychological health of college students have been affected.

## 5. Conclusions

In order to explore the physical exercise and psychological changes of college students before and after the intervention, this study adopts the method of multidimensional data mining and takes 23,146 undergraduate students from a university in Guangzhou, Guangdong Province, southern China, as research examples. This study analyzed the physical exercise and psychological changes of college students before and after the intervention, discussed the relationship between physical exercise and psychological health of college students before and after the intervention, performed an analysis of the factors affecting the physical exercise and psychological changes of college students before and after the intervention, and proposed the suggestions for improving college students' physical and psychological health under the intervention. During the intervention control period, continuous connection with others may encourage college students to actively use internal resources to actively cope with obstacles and setbacks, and as a protective factor, psychological resilience can appropriately weaken the association between risk factors in life and anxiety and relieve anxiety. Epidemiological studies have shown that physical exercise can prevent or delay the onset of various mental disorders and has the effect of single or auxiliary treatment of college students' mental illness. The results of this study shows that with the increase of age, the risk of moderate anxiety and mild depression in college students are lower; female students were more prone to mild depression than male students; college students from rural areas were more prone to mild, moderate anxiety, mild depression, and mild and severe depression than urban students; college students with nonmedical background are more likely to have moderate anxiety than those with medical background. Although some students were isolated at home and received online physical education, which urged their physical exercise to a certain extent, the intervention has hindered the opening of gymnasiums and other exercise venues, thus limiting the way college students can exercise, to a large extent affecting the physical quality of college students under the conditions. The results of this paper provide a reference for further research on the physical exercise and psychological changes of college students before and after the intervention.

## Figures and Tables

**Figure 1:** Multidimensional assessment model physical exercise and psychological changes of college students before and after the intervention based on multidimensional data mining.

**Figure 2:** Psychological changes of younger (a) and older (b) college students during the intervention.

**Figure 3:** Relationship between pass rate of psychological test and physical test of students with (a) and without (b) medical background based on multidimensional data mining.

**Figure 4:** Physical exercise and psychological changes of college students before and after the intervention based on multidimensional data mining.

**Figure 5:** Physical exercise and psychological changes of college students from rural (a) and urban (b) areas before and after the intervention based on multidimensional data mining.

**Table 1:** Sampling distribution of undergraduate students from the university in Guangzhou.

Grade	Male	Female	Medical background	Nonmedical background	Rural areas	Urban areas	Total
Freshmen	3564	2420	152	5832	4263	1721	5984
Sophomores	3522	2301	146	5677	3823	2000	5823
Juniors	3437	2286	141	5550	4011	1950	5691
Seniors	3392	2254	139	5509	3963	1685	5648
Total	13915	9231	578	22568	16060	7086	23146

**Table 2:** Statistics of psychological conduction of undergraduate students from the university in Guangzhou.

Condition	Male	Mild	Moderate	Severe	Extreme
Mental blow	254	163 (64.17%)	88 (34.65%)	3 (1.18%)	0 (0.00%)
Fear	1037	421 (40.60%)	403 (38.86%)	179 (17.26%)	37 (3.57%)
Insomnia	859	432 (50.29%)	268 (31.20%)	136 (15.83%)	23 (2.68%)
Anxiety	2748	1286 (46.80%)	1044 (37.99%)	353 (12.85%)	65 (2.37%)
Loneliness	3857	1743 (45.19%)	1395 (36.17%)	516 (13.38%)	203 (5.26%)
Self-blame	453	212 (46.80%)	141 (31.13%)	62 (13.69%)	38 (8.39%)
Hallucination	134	55 (41.04%)	47 (35.07%)	32 (23.88%)	0 (0.00%)
Irritability	3827	1692 (44.21%)	1203 (31.43%)	903 (23.60%)	29 (0.78%)
Tantrums	2236	1012 (45.26%)	624 (27.91%)	583 (26.07%)	17 (0.76%)

**Table 3:** Factors affecting the physical exercise and psychological changes of college students before and after the intervention.

Item	None	Mild	Moderate	Severe	Extreme
Concentration	+		-	+	+
Feeling	-	+	-	+	-
Temper	+	-	+	+	-
Mood	-	-	+	-	+
Figure	-	+	-	-	+
Psychology	+	-	+	+	-
Vision	+	+	-	-	-
Social contact	+	+	+		+
Learning	-	-	-	+	-
Customs	+	+	-	-	+
Physical fitness	-	-	-	-	-
Mental blow	-	+	+	-	-
Fear	-	-	+	+	-
Insomnia	+	-	+	-	-
Anxiety	-	-	+	+	-
Loneliness	-	+	+	-	+
Self-blame	+	+	+	-	+
Hallucination	-	-	-	+	+
Irritability	+	-	+	+	-
Tantrums	+	+	-	+	+

## Data Availability

The data used to support the findings of this study are included within the article.
